# A Novel U-Net Based Deep Learning Method for 3D Cardiovascular MRI Segmentation

**DOI:** 10.1155/2022/4103524

**Published:** 2022-05-20

**Authors:** Yinan Lu, Yan Zhao, Xing Chen, Xiaoxin Guo

**Affiliations:** ^1^College of Computer Science and Technology, Jilin University, Changchun 130000, China; ^2^College of Artificial Intelligence, Jilin University, Changchun 130000, China

## Abstract

Medical multiobjective image segmentation aims to group pixels to form multiple regions based on the different properties of the medical images. Segmenting the 3D cardiovascular magnetic resonance (CMR) images is still a challenging task owing to several reasons, including individual differences in heart shapes, varying signal intensities, and differences in data signal-to-noise ratios. This paper proposes a novel and efficient U-Net-based 3D sparse convolutional network named SparseVoxNet. In this network, there are direct connections between any two layers with the same feature-map size, and the number of connections is reduced. Therefore, the SparseVoxNet can effectively cope with the optimization problem of gradients vanishing when training a 3D deep neural network model on small sample data by significantly decreasing the network depth, and achieveing better feature representation using a spatial self-attention mechanism finally. The proposed method in this paper has been thoroughly evaluated on the HVSMR 2016 dataset. Compared with other methods, the method achieves better performance.

## 1. Introduction

In multiobjective segmentation, medical image segmentation aims to segment the images into multiple regions and extract the parts of interest based on the similar characteristics or single attributes of the image, such as edge contour, structure, and shape, which is of great significance for medical image analysis, disease diagnosis, and clinical applications (e.g., 3D computed tomography (CT) and magnetic resonance image (MRI)). Accurate segmentation can not only help precise diagnosis and prediction of prognosis but also benefit surgical planning and intraoperative guidance.

For example, in diagnosing congenital heart disease, segmenting the blood pool and myocardium from 3D cardiovascular magnetic resonance (CMR) images is a prerequisite before creating patient-specific heart models for preprocedural planning of children with complex congenital heart disease (CHD).

One of the main applications of deep learning is medical field, including biomedicine and MRI analysis [1]. However, the level of doctors is uneven, and some departments are labor-intensive, which has had a profound impact on the development of artificial intelligence in this field [2]. Currently, segmenting vital organs or structures from 3D medical images is an imperative preliminary action for a wide range of clinical treatments. The recognized standard segmentation results are obtained from experienced physicians and radiologists via visual inspection and manual delineations. On the one hand, there always are hundreds of images in an individual's cardiac MRI. It is tedious, time-consuming, and costly to annotate the 3D medical images in a slice-by-slice manner. On the other hand, the whole heart's manual labeling is subjective and suffers from low reproducibility. The results of the labeling could be seriously affected by the experience and knowledge of the observer. Consequently, automatic medical image segmentation with high accuracy is highly demanded. However, using deep learning for automatic medical image segmentation with high accuracy is also a huge challenge [3]. The reasons include (I) the missing borders or indefinite boundaries, with inadequate edge information, and (II) the too low quality of the cardiac images.

There are many deep learning models applied to image segmentation [4]. Convolutional neural network (CNN) based deep learning strategies especially achieved remarkable success in medical image segmentation methods. U-Net [5] is a semantic segmentation network based on fully convolutional networks (FCN) [6], which mainly applied CNN structure for the heart segmentation. U-Net can be quickly trained on small sample data in medical segmentation by data augmentation and achieve outstanding segmentation results. Different from the FCN structure, there is not any encoder or decoder in the U-Net. U-Net contains two paths, the downsampling contraction path, which extracts the high-level abstract features of pixels, and the extended upsampling path, which can reconstruct pixel information lost during downsampling. In the process adopted above, the parts from the comprehensive upsampling approach and the features extracted by downsampling are stitched to maximize the retention of low-level feature information lost by the pooling and convolution operations. Compared with FCN, U-Net can run more efficiently because there is no fully connected layer in the structure. The paper on DenseNet [7] was voted the best paper of CVPR in 2017, which has the same basic idea as ResNet [8]. However, it establishes the dense connection between all the previous layers and the latter layers. The dense block in the DenseNet is a densely connected network model between layers. In each dense block, the input of each layer is the union of the outputs of all the previous layers. DenseNet enhances feature representation with skip connections.However, the feature maps in DenseNet are relatively large, resulting in a large amount of computation in the convolution process, which affects the overall performance of the network.

This paper proposes a novel and efficient 3D sparse convolutional network named SparseVoxNet to comprehensively address these challenges, which can effectively carry out voxel-to-voxel learning and infer 3D medical images. Specifically, we develop a sparse convolutional network that aims to contribute the following ideas:

(1) The sparse network can eliminate redundant computation, reduce model parameters, and decrease the risk of overfitting small sample training data. (2) The full skip connection mechanism in the module can effectively solve the problem of gradient disappearance in 3D deep model training, accelerate the convergence speed, and improve recognition ability. (3) The self-attention mechanism is added to optimize the expression ability of feature maps and capture the long-range dependency between features better.

## 2. Related Work

Multiobjective image segmentation can be divided into supervised and unsupervised methods. Pham et al. [9] proposed a multiobjective optimization approach to segment the brain MRI using fuzzy entropy clustering and region-based active contour methods. Hongwei et al. [10] proposed a multiobjective clustering and toroidal model-guided tracking method to distinguish vascular structures from complicated structures in background regions. In recent years, deep learning has been successfully applied to medical image segmentation. Çiçek et al. [11] proposed a 3D U-Net network structure to realize the 3D image segmentation. Habijan et al. [12] proposed a framework consisting of two 3D U-Nets. In this framework, the first network was used for localizing the bounding box encompassing the heart, and the second network was employed to segment the different substructures. Ding et al. [13] incorporated attention mechanism within the gradient expanding process to enhance the coarse segmentation information with less computation expense. Furthermore, they extended the network's gradient flow and used the low-resolution feature information. Jeevakala et al. [14] proposed a Mask R-CNN approach driven with U-Net to detect and segment the Internal Auditory Canal (IAC) and its nerves. In this method, the U-Net segmented the structure related information of IAC and its nerves by learning its features.

However, the variants' structure of U-Net suffers from redundant information. More and more network structures have been proposed and applied to image analysis [15].

Fisher and Koltun [16] proposed a new convolutional network module which used dilated convolutions. This module could aggregate multiscale contextual information systematically without losing resolution. Recently, dilated convolution is increasingly applied to medical images. Wolterink et al. [17] proposed a method to segment the myocardium and blood automatically in CMR of patient who has CHD by CNN. In the same year, Fisher et al. [18] developed a convolutional network module specifically for intensive prediction which used extended convolution to systematically aggregate multiscale context information without loss of resolution. Residual network (ResNet) was proposed in 2016, which added skip connections to each convolution layer for 2D image classification tasks. In addition, this architecture has been extended to 3D volumetric segmentation [19–21]. Huang et al. proposed the DenseNet with L(L + 1)/2 direct connections, which improved ResNet. It can strengthen feature propagation and reuse all features. After this improvement, Jégou [22] proposed a 2D fully convolutional DenseNet for semantic segmentation. In the same year, Yu et al. [23] proposed the DenseVoxNet; this network extended the deep residual learning in 2D image recognition tasks into 3D, which could simplify network training, reduce the parameters, and add auxiliary paths to enhance gradient propagation. However, there were no direct connections between the dense blocks and the final prediction layer. DenseVoxNet may not be able to appropriately capture multiscale contextual information useful for accurate segmentation. The correlation of adjacent images or frames should be effectively exploited for improving the accuracy of the target tasks which involves 3D volumetric data. Therefore, more and more methods have been proposed to use 3D features for biomedical volumetric data [24–29]; for example, Hosseini-Asl et al. [30] proposed a deep supervised adaptive 3D CNN, which could automatically extract and recognize the characteristics of Alzheimer's disease and capture the changes caused by Alzheimer's disease, such as the size of ventricle, the shape of the hippocampus, and the thickness of cortex. Dou et al. [31] proposed a 3D fully convolutional network, called 3D Deeply Supervised Network (DSN), equipped with a deep supervision mechanism. This method has obtained good results in two tasks: liver segmentation of 3D CT scan, and whole heart and large blood vessels segmentation of 3D MRI. Previous CNN expresses dependencies between different image regions through convolution. Convolution operators have local receptive fields, so processing long-range dependencies goes through multiple convolutional layers, which may prevent learning about long-term dependencies. While it is possible to increase the representational capacity of the network by increasing the size of the convolutional kernels, the computational and statistical efficiency gained by using local convolutional structures are lost. However, self-attention [32–34] can exhibit a better balance between the ability to model long-range dependencies and computational efficiency. However, it is still a challenging task for CNNs to segment the important organs from 3D medical images due to the complexity of 3D structures, the difficulty of voxelized grid optimization, and the insufficiency in training samples.

Dou et al. [35] proposed Pnp-AdaNet using the method of adversarial learning, which could adapt to medical images of different modalities through plug-and-play modules. In another experiment, Dou et al. [36] constructed a domain adaptation module (DAM) to map the target region to features that were spatially aligned with the source domain region. The domain critic module(DCM) was responsible for distinguishing the feature spaces of the two domains. Then these two modules were optimized via an adversarial loss without using any target domain label. They trained the network using MRI, used it to segment CT images, and finally achieved certain results. The experiments done by Schlemper et al. [37] showed that using a grid-like attention mechanism in CT images might achieve better results. Shi et al. [38] proposed Bayesian VoxDRN for segmenting the entire heart from 3D MRI. Bayesian VoxDRN could predict voxel class labels by measuring the uncertainty of the model. During the test, it was realized by sampling based on Monte Carlo to generate a posteriori distribution of voxel labels. The attention mechanism was first applied to the text field. When the improved attention mechanism was applied to image processing, very good results were achieved. Liu et al. [39] proposed a novel medical image super-resolution method based on dense neural network and blended attention mechanism to address the problem that medical image would suffer from severe blurring caused by the lack of high-frequency details in the process of image super-resolution reconstruction. Kaul et al. [40] joined the attention tool to CNNs using feature maps generated by a separate convolutional autoencoder. This attention architecture was well suited for incorporation into deep convolutional networks. The results showed that this attention architecture was better than U-Net and residual variant.

## 3. Methods

### 3.1. The Architecture of SparseVoxNet

The architecture of SparseVoxNet proposed in this paper is shown in Figure 1. It improves U-Net which includes upsampling and downsampling processes to implement end-to-end training. The padding is used for keeping the feature-map sizes constant in every sparse block, because the sparse block is not applicable when the feature maps have different sizes. Therefore, in each sparse block, the first 4 layers use ordinary convolutions, and the last 3 layers use dilated convolutions. The hole sizes are 2, 3, and 5. The spatial self-attention mechanism is added after the original feature map of data to strengthen the more important features in the original feature map. In the final deconvolution layer, instead of using a fully connected layer, three 1 × 1 × 1 convolution layers and softmax layer are used to obtain the segmented final label map. A dropout layer with a coefficient of 0.2 is added after each convolution layer to enhance the generalization ability of network.

Inspired by DenseNet, the black dotted line in SparseVoxNet in Figure 1 represents a skip connection. The image is segmented once by deconvolution on the skip connection. The network will converge faster and the accuracy rate will be higher due to the skip connection. The first segmented image will perform better on edge segmentation, because the shallow neural network loses less information through convolution and gets more edge information. The result is a fine grained segmentation. The result of the second segmented image is better in overall segmentation, which is coarse grained segmentation. Deep neural network features are high-level abstract features, which is really helpful when extracting the segmented central area of the entire tissue. The final segmentation result is determined by the voting of multiple segmentation results of different cropped input data on a single voxel point. The downsampling process of U-Net is replaced with sparse blocks, and the two deconvolutions are equivalent to the upsampling process.

Furthermore, we calculate the number of parameters for each layer in the SparseVoxNet shown in Table 1. Table 1 shows the parameters of 4 convolution layers, 2 deconvolution layers, 2 sparse blocks, a spatial attention mechanism layer, and a skip connection layer. Among them, the 4 convolution layers are represented by Conv_n, the 2 deconvolution layers are represented by Deconv_n, and the 2 sparse blocks are represented by Sparse Block_n. We also show the convolution kernel and stride of each layer in Table 1. Note that each row in Table 1 corresponds to each layer in Figure 1.

### 3.2. Sparse Block

DenseNet has denser connections compared to ResNet, which makes the consumption of hardware resources very high. Therefore, we propose a sparse network structure to change the way of feature reuse while keeping feature reuse and skip connection characteristics unchanged. The sparse block which we propose reduces the number of connections, just having direct connections between any two layers with the same feature-map size, referred to as full skip connection, but the effect of sparse block is similar to dense block. The input of transition layer is as follows:

(1) $$\begin{array}{c} \left[T_{0},T_{1},T_{2},T_{3},T_{4}\right]=\left[T_{0},H_{1}\left(T_{0}\right),H_{2}\left(T_{1}\right),H_{3}\left(T_{2}\right),H_{4}\left(T_{3}\right)\right]. \end{array}$$

where the input of *H*_1_ is *T*_0_, the input of *H*_2_ is *T*_0_ + *T*_1_, and so on.

The feature maps of different receptive fields are referred to as different scales. It is found that the nonlinear combination of the features of different scales is not better than the linear combination. Inspired by the U-Net network structure, composite expression features are constructed by directly stacking feature maps of different scales.

Unlike U-Net, the improved network structure uses deconvolution to replace the upsampling process, which reduces the loss of information during the conversion process. In DenseNet, the network connections of the previous layer and the latter layer are too dense, which can easily cause overfitting. The sparse network can solve this problem. The network's feature expression ability is greatly enhanced, and there is no vanishing gradient.

### 3.3. 3D Dilated Convolution

Dilated convolution has one more hyperparameter than traditional convolution, called dilation rate. Dilated convolution adds holes to the standard convolution kernel. In this paper, we extend the dilated convolution to 3D data, and mix the traditional convolution and dilated convolution. Referring to the DenseVoxNet, we use 4 layers of 3 × 3 × 3 traditional convolution and 3 layers of dilated convolution with 2, 3, and 5 holes. The 4 layers of traditional convolution can extract the local features of the image, and the 3 layers of dilated convolution expand the reception field of the feature exponentially to capture the potential relationship between long distance features. We only use 7-layer convolution to make the reception field reach 26 × 26 × 26.

### 3.4. Spatial Self-Attention Mechanism

In both the computer vision tasks and the natural language processing tasks, the dependencies between long distance features are difficult to capture. In serialization tasks, recurrent and recursive neural networks are major means to capture long-range dependencies. In convolutional neural networks, large reception fields are formed by superposing multiple convolution operations. Currently, there are no specific methods to capture long-range features. Convolution and cyclic operators have the following disadvantages: (1) being too inefficient, (2) easily producing gradient disappearance, (3) difficulty of passing information back and forth between long ranges.

Inspired by the nonlocal mean filtering for images, Wang et al. [41] proposed nonlocal block for capturing long-range dependencies, which is a self-attention mechanism. Nonlocal block ignores the Euclidean distance and calculates the relationship between two positions directly. Actually, it calculates the generalized autocorrelation matrix of features. However, the calculation efficiency is relatively high. Because after adding nonlocal operators, it is not necessary to stack too deep convolution operations for achieving the network's fitting ability. Furthermore, it does not change the size of input data and can be easily embedded in the network, so the spatial self-attention model is added in front of the first sparse block. We apply the self-attention mechanism, proposed by Zhang et al. [42], in this paper. The nonlocal block is embedded in the 3D network, which is defined as follows:

(2) $$\begin{array}{c} y_{i}=\frac{1}{C\left(x\right)}\sum_{\forall j}f\left(x_{i},x_{j}\right)g\left(x_{j}\right)\text{,} \end{array}$$

where *i* is a 3D coordinate meaning the position index of input data, *j* is the index of all possible positions, *x* is the input data, *f* is an autocorrelation calculation function, which can calculate the correlation between *i*-th position and *j*-th position, and *g* is a unary mapping function. The 1 × 1 × 1 convolution is used for ascending dimension and fusing the multichannel feature in the experiments, and finally *C* (*x*) is used for normalization. Using multiple 1 × 1 × 1 convolution kernels in the attention model can not only achieve cross-channel interaction and information integration, but also reduce or increase the number of channels. People begin to pay attention to the 1 × 1 × 1 convolution because of the network structure proposed by Lin [43]; this convolution connects two full connection layers for fusing the features linearly. After that, in Google's Inception-v4 [44] network structure, 1 × 1 × 1 convolution is used in the inception module for dimensionality reduction or ascending dimension. Inspired by this advantage, in this paper, the 1 × 1 × 1 convolution kernel is used to reduce the original input data dimensionality, calculate the spatial autocorrelation relationship, and then ascend the dimension of data. The different weights calculated are added back to the original data and then regularized to describe the influence on features of voxel points in different spatial positions.

## 4. Experiments and Results

### 4.1. Dataset

Radiobiological images mainly have six data formats. The NIFTI (Neuroimaging Informatics Technology Initiative) is one of them. The data format used in this paper is NIFTI. This format contains two affine coordinates, so that it can associate the physical index of voxels with its actual spatial location. The HVSMR 2016 dataset is used to evaluate the algorithm and network structure. HVSMR 2016 has a total of 10 cardiac magnetic resonance 3D scans for training and 10 scans for testing. All training sets of cardiac MRIs are from patients with CHD, including annotations of myocardium and large blood vessels.

Due to the large difference in intensity between different images, the cardiac MR images are all normalized. After normalization, the mean and unit variance are 0. To leverage the limited training data, simple data augmentation was employed to enlarge the training data. The augmentation operations include the rotation and cropping. The original training set is divided into three parts, namely, the training set, the validation set, and the testing set. The cross-validation method is used for parameter training. We use 70% of the images for training and 30% for testing. Then, we compare and briefly discuss the experimental results. 

### 4.2. Evaluation Metrics

Medical image segmentation is an important step of medical image processing. However, it is difficult to select accurate evaluation index to evaluate the quality of segmentation by comparing segmented medical images. The following three metrics are used in this paper for measuring the results of segmentation.

#### 4.2.1. Dice Coefficient

Dice coefficient is widely used for verifying the effect of 3D medical image segmentation. The core idea is to ensure a high recall and precision. Compared with the evaluation method of directly computing the difference between the automatic segmentation results and the original data labels, using Dice coefficient can better characterize the segmentation effect. Dice coefficient is defined as follows:

(3) $$\begin{array}{c} \text{Dice}=\frac{2\left|G\cap R\right|}{\left|R\right|+\left|G\right|}=\frac{2\text{TP}}{2\text{TP}+\text{FP}+\text{FN}}\text{,} \end{array}$$

where *G* is the segmentation result of ground truth, which is the labeled testing data. *R* is the automatic segmentation result of testing data. TP, FP, and FN represent true positives, false positives, and false negatives, respectively, for each class. Ideally, the template of segmentation result and the template of label data completely overlap, which means *R* = *G*, and the absolute value of the Dice coefficient is 1.

#### 4.2.2. Average Symmetric Surface Distance

Average symmetric surface distance (ADB) is defined as follows: for a single voxel point, if one or more voxel points within its 18-neighborhood are not elements of the object, they are regarded as surface voxel points. For each surface voxel point in the *R*, we calculate the Euclidean distance between it and the nearest surface voxel point of the real label *G*. Similarly, perform the same calculation for each surface voxel point in the *G*. *S* (*R*) represents the surface voxel point set of *R*. The distance from any voxel point v to *S* (*R*) is defined as $d\left(v,S\left(R\right)\right)=\underset{s_{R}\in S\left(R\right)}{\min}\left|\left|v-s_{R}\right|\right|$. Based on this formula, the average symmetrical surface distance is defined as follows:

(4) $$\begin{array}{c} \text{ADB}=\frac{1}{\left|S\left(G\right)\right|+\left|S\left(R\right)\right|}\times \left[\underset{s_{R}\in S\left(R\right)}{\sum }d\left(s_{R},S\left(G\right)\right)+\underset{s_{G}\in S\left(G\right)}{\sum }d\left(s_{G},S\left(R\right)\right)\right]. \end{array}$$

Many segmentation boundary evaluation metrics are constructed based on this distance formula, which measures the boundary difference between the segmentation result and the ground truth by calculating the voxel surface distance. The larger the value of ADB, the more dissimilar the segmentation boundary is. When the boundary of the segmentation result matches the ground truth exactly, the value of ADB is 0.

#### 4.2.3. Hausdorff Distance

Based on the ADB, when using the maximum symmetric distance, the metric is known as Hausdorff distance, which is defined as follows:

(5) $$\begin{array}{c} \text{hausdorff}\left(R,G\right)=\underset{r\in R}{\max}\left\{\underset{g\in G}{\min}\left\{d\left(r,g\right)\right\}\right\}, \end{array}$$

where *d* (*r*, *g*)  represents the distance between points *r* and *g*; that is, the set consists of the shortest distance (usually expressed in Euclidean distance) from all points in the predicted segmentation set *R* to any point in the real label set *G*, and the maximum distance is selected from this set as the Hausdorff distance between the two sets *R* and *G*. This distance and the symmetrical surface distance both describe the similarity of the contour. The larger the absolute value, the less similar the segmentation.

### 4.3. Training

In the experiments, all weights are randomly initialized by the Gaussian distribution with *μ* = 0, *θ* = 0.01, and the stochastic gradient descent optimization algorithm is used. Batch size is set to 8. In order to reduce the model overfitting and speed up the convergence rate, the weight attenuation is 0.0005, and the momentum is set to 0.9, which is often used to speed up training, while making it easier to jump out of extreme points and avoid getting stuck in local optimal solutions. The drop rate is 0.2, and the initial learning rate is set to 0.01. If the learning rate is too low, the training period is too long, and the high learning rate will cause the model to be unstable and never converge. Our algorithms were trained and tested on the Dual RTX 2080 Ti GPU.

The polynomial decaying learning rate is used for ensuring the rapid convergence of the model during the initial training period and the stability of the model parameters in the later period. The initial learning rate is set relatively large, and the learning rate is reinitialized and decayed every 5000 steps. The attenuation coefficient of the learning rate is *δ*=(1 − iter/max_iter)^power^. After testing, the model stabilizes after 8000 iterations. The input data of SparseVoxNet consists of 8 groups of 64 × 64 × 64 heart MRIs, which are cropped randomly in the same axis direction.

Multiple sets of comparative experiments and ablation experiments are designed to verify the effect of the improved method on segmentation. In the experiments, we compared our method with the traditional methods and other deep learning methods, and also compared the network only with the mixed dilated convolution and the network only with the attention mechanism and DenseVoxNet. 

#### 4.3.1. Ablation Study

We conduct ablation experiments to verify the importance of 3D dilated convolution and spatial self-attention mechanism in exploiting multiscale features. The results are presented in Table 2.

When we just add the mixed 3D dilated convolution to the model, we define this model as SparseVoxNet-D. The Dice coefficient of myocardium and blood pool gets the best results, 82.4% and 91.6%, respectively. It verifies our conjecture: dilated convolutions can exponentially expand receptive fields to obtain multiscale information without losing resolution or coverage, especially for structures with a small size or irregular boundary, such as the cardiac myocardium structures. Since the receptive field expansion speed of the dilated convolution depends on the number of holes in the dilated convolution, although the more holes will contribute a larger receptive field, the pixels in the large receptive field are not necessarily related to the current convolution. In other words, the larger receptive field is not the better. Local perception can better capture local features. Global perception can better capture the relationship characteristics of pixels at different locations. Hence, we mix the 4 layers of traditional convolution and 3 layers of dilated convolution and define the different dilation rates of dilated convolutions to better capture features.

When we just add the spatial self-attention mechanism to the model, we define this model as SparseVoxNet-S. It can be seen that ADB and Hausdorff distance of blood pool and myocardium achieve better performance than DenseVoxNet, the Hausdorff distance of myocardium outperforms DenseVoxNet by around 3.0%, and the Hausdorff distance of blood pool outperforms DenseVoxNet by around 4.8%. This indicates that with the spatial self-attention mechanism, the segmented images have been brought closer to the target domain successfully, because the self-attention in our model is complementary to the convolution for capturing long-range, global-level dependencies occurring in cardiac structure. The advantages of the attention mechanism are as follows: (a) few parameters; (b) fast calculation; (c) capturing long-range features. The problem applied in this paper is a small sample training process, so when the spatial self-attention mechanism is removed, the segmentation result is not ideal, which means the long-range features cannot be extracted efficiently. We use both dilated convolution and spatial self-attention mechanism to capture long-range features, because the method based on dilated convolution obtains information from a small number of surrounding points and cannot form dense context information. The spatial self-attention mechanism makes a single feature in any location perceive the features of all other locations, and can produce more powerful pixel-level representation capabilities. These observations demonstrate that the 3D dilated convolution and the spatial self-attention indeed play a meaningful role in exploiting multiscale features.

### 4.4. Results

There are segmentation results on three training images shown in Figure 2. These three slices come from different patients. The data whose indexes are 60 in the sample dataset have the same coronal plane view in the same dimension. The light blue and dark blue areas of the image in the first line represent the blood pool and myocardium; the dark blue and black areas belong to the background. The images in the second line are labeled, corresponding to the myocardium and blood pool in the first line of images. The third line is the results of automatic segmentation by the method proposed in this paper, where blue, yellow, and dark purple represent the myocardium, blood pool, and background, respectively. It can be seen from Figure 2 that although the cardiac structure of different patients in the training set is quite different, the method we proposed can still successfully calibrate the myocardium and blood pool from low contrast cardiac MRI, which proves that this method has a good enough fitting ability to the original data. However, there are still some disadvantages. In the first auto-segmentation result, the myocardium in the lower left corner is partially divided. In the second result, the background appeared in the myocardium. In the third result, there is extra myocardium in the upper right corner, which shows that deep learning has the ability to perceive most data features, but it does not have reasonable logical reasoning capabilities. Human segmentation will not produce these subtle logical errors.

Figure 3 shows segmentation results on three testing images. The data extraction method is the same as above. By observing the results, we can see that the method proposed in this paper also has good generalization effect on unlabeled data. However, when using the gradient descent algorithm, it is easy to fall into the local optimum and cause overfitting, because of the huge number of parameters.

### 4.5. Discussion

The comparison of the results between the method we proposed and other six methods is shown in Figure 4. They are mainly ranked according to the Dice coefficient. The figure also shows the auxiliary reference indexes, such as ADB and symmetric Hausdorff distance. The first three are traditional methods, such as manually extracting features and using hidden Markov random fields, and the other deep learning methods are on the HVSMR 2016 Challenge dataset. According to Figure 4, the Dice coefficient of blood pool in all methods is higher than that of myocardium, suggesting that the segmentation of blood pool is relatively easier due to the ambiguous borders of the myocardium in the low-resolution MRIs. Regarding the segmentation of myocardium, the method we proposed achieves the best performance with the Dice; i.e., the ranking metric in the challenge, 0.861 ± 0.024, outperforms the second one by around 4%. The best result also has been achieved in blood pool segmentation with Dice; the ranking metric in the challenge, 0.94 ± 0.016, demonstrates that our sparse connected network has the capability to tackle hard cardiovascular segmentation problem. The ADB and Hausdorff distance of our method also achieved the best performance.

The results of other 3D MRI segmentation methods are mainly shown in Table 3. Firstly, the experimental parameters are compared, and the method proposed in this paper needs the least parameters. The sparse block and dilated convolution can achieve a good fitting effect with the participation of such a small number of parameters, thanks to the introduction of the attention model. The feature expression ability of sparse block will not be better than dense block in many cases, but the problem applied in this paper is medical segmentation and a small sample training process, so the sparse block can fit and generalize the data well with a small number of parameters, and the exponentially increasing receptive field provided by the dilated convolution reduces the convolution operations. The attention mechanism can well capture the features to strengthen the generalization ability of the network. Because of the small number of parameters, the amount of calculation is reduced, and the model's convergence rate is also fast.

Comparing the cross-entropy loss of DenseVoxNet and SparseVoxNet with sparse block and dilated convolution, we can find that the network only using the mixed dilated convolution can converge faster and reach lower loss values, which proves that the improved sparsely connected network structure can reduce the calculation amount and improve the efficiency and that the method of extracting long-range features by hybrid 3D dilated convolution is suitable for medical images. It has better ability to represent features and fit data .

The comparison shows that the time of one iteration of DenseVoxNet (forward and backward propagation of the network) is 0.113 s, the time of SparseVoxNet-D is 0.045 s, and the time of SparseVoxNet is 0.049 s. The proposed method has a great improvement in efficiency.

## 5. Conclusion

In this paper, we propose a novel and efficient 3D sparse convolutional network to segment blood pool and myocardium from 3D cardiac magnetic resonance images. This method can eliminate redundant calculations and reduce model parameters and the risk of overfitting training data on small samples. The spatial self-attention mechanism can optimize the expression ability of feature maps, and the sparse blocks can reduce the convolutional network depth. The work in this paper is an accurate pixel-level classification. Moreover, we achieve competitive results in comparison with existing methods. The proposed method can provide comprehensive information for doctors to make diagnoses of CHD.

## Figures and Tables

**Figure 1:** An overview of the proposed SparseVoxNet, with intermediate feature volumes. The light blue and dark blue areas of the slice represent the blood pool and myocardium. The dark blue and black areas belong to the background. The blue, yellow, and dark purple of segmented result represent the myocardium, blood pool, and background, respectively. There are two sparse blocks in this network. The black dotted line at the bottom right represents a skip connection.

**Figure 2:** Segmentation results on three training images.

**Figure 3:** Segmentation results on three testing images: The three slices in the first line come from different patients. Images in the second line are the results of automatic segmentation by the method proposed in this paper.

**Figure 4:** Comparison of experimental results between the improved method and other methods.

**Table 1:** Our 3D convolutional model.

Input image				Output				Layer (type)	Stride	Kernel	Parameters
64	64	64	1	32	32	32	16	Conv_1 (convolution)	2	3	448
32	32	32	16	16	16	16	16	Conv_2 (convolution)	2	3	6928
16	16	16	16	16	16	16	16	Spatial attention	2	1	816
16	16	16	16	16	16	16	100	Sparse Block_1 (sparse block)	1	3	43300
16	16	16	100	16	16	16	100	Conv_3 (convolution)	1	1	10100
16	16	16	100	16	16	16	184	Sparse Block_2 (sparse block)	1	3	496984
16	16	16	184	16	16	16	64	Conv_4 (convolution)	1	1	11840
16	16	16	64	32	32	32	64	Deconv_1 (deconvolution)	2	4	262208
32	32	32	64	64	64	64	64	Deconv_2 (deconvolution)	2	4	262208
16	16	16	100	64	64	64	64	Skip connection	1	1	6464

**Table 2:** Results of ablation study. Bold results are the best ones.

	Myocardium			Blood pool		
Method	Dice (%)	ADB	Haus.	Dice (%)	ADB	Haus.
SparseVoxNet-D	**82.4**	0.922	5.385	**91.6**	1.073	7.736
SparseVoxNet-S	80.7	**0.853**	**5.075**	91.4	**0.951**	**5.004**
DenseVoxNet	79.2	0.943	7.175	89.48	0.955	9.608

**Table 3:** Comparison of experimental results between the improved method and the 3D methods. Bold results are the best ones.

	Myocardium			Blood pool		
Method	Dice (%)	ADB	Haus.	Dice (%)	ADB	Haus.
3D U-Net [11]	69.4	2.596	12.796	79.4	2.550	14.634
V-Net [26]	70.3	2.367	10.624	81.9	2.435	12.539
VoxResNet [19]	77.4	2.041	13.199	86.7	2.157	19.723
DenseVoxNet [23]	79.2	0.943	7.175	89.48	0.955	9.608
Ours	**84.5**	**0.721**	**5.027**	**94.0**	**0.831**	**4.102**

## Data Availability

The data used in this study could be accessed upon request.
